The article "Short-Term Demand Forecasting Method in Power Markets Based on the KSVM–TCN–GBRT" was published in 2022. Journal: Comput Intell Neurosci.

# Short-Term Demand Forecasting Method in Power Markets Based on the KSVM–TCN–GBRT

**DOI:** 10.1155/2022/6909558

**Published:** 2022-04-30

**Authors:** Guang Yang, Songhuai Du, Qingling Duan, Juan Su

**Affiliations:** College of Information and Electrical Engineering, China Agricultural University, Beijing, China

## Abstract

With the consumption of new energy and the variability of user activity, accurate and fast demand forecasting plays a crucial role in modern power markets. This paper considers the correlation between temperature, wind speed, and real-time electricity demand and proposes a novel method for forecasting short-term demand in the power market. Kernel Support Vector Machine is first used to classify real-time demand in combination with temperature and wind speed, and then the temporal convolutional network (TCN) is used to extract the temporal relationships and implied information of day-ahead demand. Finally, the Gradient Boosting Regression Tree is used to forecast daily and weekly real-time demand based on electrical, meteorological, and data characteristics. The validity of the method was verified using a dataset from the ISO-NE (New England Electricity Market). Comparative experiments with existing methods showed that the method could provide more accurate demand forecasting results.

## 1. Introduction

The inherent volatility and uncertainty of renewable energy sources, such as wind power and photovoltaics, may lead to large deviations between the bid output and the actual output when renewable energy sources participate in the market. Also, customers change their electricity load when they receive a price change or incentive signal from the supply side, taking into account their own production or consumption. Hence, timely and accurate information on the demand changes has imposed higher requirements on the accuracy of demand forecasting [1].

In current electricity forecasting, it is necessary to fully integrate economic, meteorological, and other multidimensional information; use advanced data-driven processing means; and deeply analyze the change patterns and laws of renewable energy and demand [2]. This creates the need to study demand response characteristics under multidimensional variables in the electricity market environment to improve forecasting accuracy [3]. For power system operation, short-term demand forecasts can predict demands from 1 hour to 168 hours in advance [4]. To obtain accurate forecasting results, different forecasting models such as regression, statistical, and state-space methods are used. Expert system-based, evolutionary process, fuzzy systems, and artificial intelligence algorithms have also been introduced. Wang et al. [5] proposed a method that decomposes the demand into the trend series and the fluctuating series and then builds the corresponding forecasting models separately. To improve the internal clustering performance, Dongyeon et al. [6] proposed the logistic mixed vector autoregression model, which combines clustering and prediction into one model through an expectation-maximization algorithm. Dong et al. [7] proposed an indicator variable to capture the abnormal information on special days, such as national holidays, proximity days, and bridging days. In Yin et al. [8], the multispatiotemporal convolutional network was applied to short-term demand prediction tasks, which reduced the noise error of demand data and enhanced the time-series characteristics of demand data. In [9], the demand was decomposed into different frequency components using an integrated empirical modal decomposition algorithm; the low-frequency components were then predicted using multivariate linear regression, the high-frequency components were predicted using a long short-term memory neural network (LSTM), and the components were finally combined to obtain the demand forecast. Han et al. [10] presented a short-term individual residential demand forecasting model based on a combination of deep learning and k-means clustering, which is capable of effectively extracting the similarity of residential demand and performing residential demand forecasting accurately at the individual level. It first makes full use of k-means clustering to extract the similarity among residential demand and then employs deep learning to extract complicated patterns of residential demand. Lv et al. [11] designed a LightGBM-optimized LSTM to realize short-term stock prices. To improve the demand prediction accuracy in the case of single sample data, Mei et al. [12] proposed a model based on multiscale temporal features for LSTM. First, wavelet decomposition decomposes historical data into stable components, trend demand, and periodic series such as the response peak-valley magnitude and duration, highlighting different time-scale features. Second, LSTM is used to achieve further extraction of time-series characteristics and data fitting. Finally, the model directly outputs predicted values for multiple moments. M. Hadi Amini et al. [13] proposed an autoregressive integrated moving average method for forecasting conventional electrical loads and electric vehicle parking charging demand. Kianoosh et al. [14] proposed to model the nonseasonal and seasonal cycles of load data using regression (AR) and moving average (MA) components, which have been used to forecast electricity demand at different time scales. Moreover, Zhang et al. [15] used Singular Spectrum Analysis (SSA) to preprocess the data and then used a support vector machine (SVM) optimized by the cuckoo search (CS) algorithm to model the resulting sequence with different prediction strategies. Salah et al. [16] used wrapper and embedding feature selection methods to select the optimal features and a genetic algorithm (GA) to find the optimal time lag and number of layers to optimize the predictive performance of the LSTM model, which was used to construct a short-to-medium-term cumulative load forecasting model. LU et al. [17] proposed a hybrid model short-term load forecasting method based on the convolutional neural network (CNN) and LSTM network. The CNN was first used to extract the feature vector, and the feature vector was constructed in a time-series sequence and used as the input data for the LSTM network. In [18], a convolutional long- and short-term memory network (Conv-LSTM) was proposed for electrical load data, and it achieved better accuracy than the traditional prediction algorithm based on linear regression. CHEN et al. [19] derived the respective predictions based on LSTM and LightGBM training. The optimal weighting combination method was used to determine the weighting coefficients and derive the prediction values of the combined model to improve the accuracy of load prediction. In [20], predictions were extrapolated by calculating correlations between potential variables and outputs and predicting the future consumption of high performance. In [21], a hybrid method combining empirical mode decomposition (EMD), particle swarm optimization (PSO), and a fuzzy inference system based on the adaptive network (ANFISs) for short-term load prediction of microgrids was proposed. In [22], sample entropy was used to identify the nonlinearity and uncertainty of the original time series, and the optimal mode of the original series and the optimal input form of the model were determined by the feature selection method. Finally, the least square SVM adjusted by the multiobjective sines and cosines optimization algorithm was used to predict the power demand sequence. In [23], the parameters of the LSTM were first optimized using the Sparrow Search Algorithm (SSA); then, the dataset was preprocessed, and finally, the processed data were used for residential load training and prediction. Li et al. [24] combined LSTM with quantile regression to generate multiple quantile results and introduced a combinatorial layer that considers the constraint relationships between quantile prediction values to ensure that the quantile prediction values are reasonable.

The article "Short-Term Demand Forecasting Method in Power Markets Based on the KSVM–TCN–GBRT" was published in 2022. Journal: Comput Intell Neurosci.

The TCN was proposed in 2018 to offer greater performance advantages over recurrent neural networks (RNNs) in temporal data processing tasks [25]. Following the motivation above, we propose a novel method based on Kernel Support Vector Machine (KSVM)–TCN–Gradient Boosting Regression Tree (GBRT) for improving the short-term demand forecasting accuracy of power markets. The contributions of this paper are as follows:

1. The KSVM is used to extract and train classification features for real-time electricity demand on historical data by the features of temperature and wind speed, and a numerical calculation method is used to automatically select the parameters of the KSVM to derive a classification sequence of real-time electricity demand for future days as the feature sequence.
2. A multivariable TCN method is used to capture the fluctuation trend of day-ahead demand in the day-ahead market to predict the real-time demand series in the real-time market.
3. The TCN–GBRT method integrating time-domain processing, integrated learning, and parallel feature processing is proposed. TCN is able to extract features and temporal relationships owing to its residual network and convolutional structure, avoiding gradient disappearance and gradient explosion in deep learning. GBRT can combine multiple weak classifiers into a single strong classifier that takes the best of all the weak classifiers and achieves optimal performance.

## 2. Materials and Methods

### 2.1. KSVM Model

In this paper, a Gaussian Kernel SVM is used in data feature extraction to solve the classification problem of the presence of nonlinear separability. That is, given a training sample set *D*={(*x*_1_, *y*_1_), .(*x*_2_, *y*^2^),…, (*x*_*m*_, *y*_*m*_)}, *y*_*i*_={−1+1}, the basic type of Kernel SVM is defined as in the following equation:

(1) $$\begin{array}{c} \underset{w,b}{\min}\frac{1}{2}{\left\|\omega \right\|}^{2},\\ \text{s.t. }y_{i}\left(\omega^{T}\phi \left(x_{i}\right)+b\right)\geq 1,\;i=1,2,\ldots ,m,\\ \gamma =\frac{{\left\|\omega \right\|}^{2}}{2}, \end{array}$$

where *γ* is the sum of the distances from the support vector to the hyperplane, called the “margin.” Finding the maximizing interval is equivalent to finding the minimum ||x||^2^. *ω = (ω*_*1*_*; ω*_*2*_*; …; ω*_*d*_) is the normal vector of the hyperplane, *b* is the displacement term, and *ϕ*(*x*) denotes the feature vector after mapping *x*.

The dual problem is defined in the following equation:

(2) $$\begin{array}{c} \underset{\partial }{\max}\sum_{i=1}^{m}\partial_{i}-\frac{1}{2}\sum_{i=1}^{m}\sum_{j=1}^{m}\partial_{i}\partial_{j}y_{i}y_{j}\phi {\left(x_{i}\right)}^{T}\phi \left(x_{j}\right),\\ \text{s.t. }\sum_{i=1}^{m}\partial_{i}y_{i}=0,\;\partial_{i}\geq 0,\;i=1,2,\ldots ,m. \end{array}$$

Here, *κ*(.,.) is the kernel function given in

(3) $$\begin{array}{c} \kappa \left(x_{i},x_{j}\right)=\phi {\left(x_{i}\right)}^{T}\phi \left(x_{j}\right). \end{array}$$

The kernel function maps the data from the original space into a high-dimensional Hilbert space, where a more efficient classification hyperplane exists than in the original space.

The article "Short-Term Demand Forecasting Method in Power Markets Based on the KSVM–TCN–GBRT" was published in 2022. Journal: Comput Intell Neurosci.

Suppose that {*x*_*j*_^(*i*)^}_*j*=1⋯*Ni*_ ⊂ *R*^*d*^ is the set of training samples in class *i*, where *N*_*i*_ represents the training samples in class *i* (*i*=1,2,…, *L*). The Gaussian Radial Basis Function (RBF) kernel is defined as in the following equation:

(4) $$\begin{array}{c} \kappa \left(x,z,\sigma \right)=\exp\left(-\frac{{\left\|x-z\right\|}^{2}}{2\sigma^{2}}\right),\;\sigma \in \left(0,\infty \right), \end{array}$$

where *x*, *z* ∈ *R*^*d*^, and *σ* ∈ *R* − {0} are the corresponding parameters.

### 2.2. TCN Model

TCN is a one-dimensional full convolution network, which combines the structure of causal convolution, extended convolution, and the residual network. Causal convolution means that the output time is convolved only with the elements of the previous layer of time, which ensures that there will be no information leakage in the future. Dilated convolution is designed to capture a sufficiently long history of information, and the depth of the network model increases dramatically.

Define the one-dimensional sequence input *X*(*x*_1_, *x*_2_ … *x*_*s*_), where *F* : ·{0,1,…, *k* − 1} is the function to the dilatative convolution, and the TCN convolution operation is defined as in the following equation:

(5) $$\begin{array}{c} F\left(s\right)=\left(X{\text{Con}}_{d}f\right)\left(s\right)=\sum_{i=0}^{k-1}f\left(i\right)x_{s-d\cdot i}, \end{array}$$

where *Con* is the convolution operation; *d* is the dilatative convolution parameter; *s* is the current number of sequences; *k* is *Con* Size; s-*d·i* is past directions; and a convolution with parameter *d*=1,2,4 and size *k*=3 is shown in Figure 1.

As shown in Figure 2, the mezzanine mapping is within the residual connection, as shown in equation (6). The residual network fits several nonlinear layers between the input and output data. The more the features that are extracted, the closer the residual *F*(*x*) is to 0. Hence, when the network reaches an optimal structure, *F*(*x*) is pushed to 0 as the network layers deepen, leaving only the identity mapping *x*. This overcomes the problem of TCN degradation due to increasing network layers. Using the residuals, each order of derivative plus the constant term 1 is as in equations (6) and (7). The error can still be effectively backpropagated at this point, even if the derivatives ∂*f*/∂*x* are small.

(6) $$\begin{array}{c} o=F\left(x\right)+x, \end{array}$$

(7) $$\begin{array}{c} \frac{\partial h}{\partial x}=\frac{\partial \left(f+x\right)}{\partial x}=1+\frac{\partial f}{\partial x}, \end{array}$$

where *F(x)* is a residual function; *x* is a constant.

The article "Short-Term Demand Forecasting Method in Power Markets Based on the KSVM–TCN–GBRT" was published in 2022. Journal: Comput Intell Neurosci.

### 2.3. GBRT Model

The GBRT algorithm is able to compensate for the tendency of the cart algorithm to overfit small sample data or produce instability and low prediction accuracy. The algorithm is an iterative decision tree algorithm, which consists of three parts: cart, Gradient Boosting algorithm, and reduction idea.

The basic idea of the algorithm is to use the Boosting method to iterate multiple weak learners with low prediction accuracy to form a strong learner with high prediction accuracy, that is, to reduce the residuals of the previous model by learning again so that the next generated model has a smaller error. The gradient iteration makes the combined model continuously improved, which is a kind of decision tree integrated learning algorithm designed to improve the model learning rate and prevent overfitting. That is, it does not fully trust each residual tree and uses gradual approximation to learn through multiple tree residuals.

For continuous data types, the loss function is the classical loss function in Boosting, that is, the sum of squared errors, which is calculated as shown in (4). After *M*-th iterations, the prediction is shown in equations (8) and (9).

(8) $$\begin{array}{c} L\left(y,f\left(x\right)\right)=\sum_{i=1}^{n}{\left(y_{i}-f\left(x_{i}\right)\right)}^{2}, \end{array}$$

(9) $$\begin{array}{c} f\left(x\right)=\sum_{i=0}^{n}f_{i}\left(x\right), \end{array}$$

where *x* is the input variables, *y* is the output variables, and *i* is the iteration count.

The key to improving the prediction accuracy of the GBRT model is the calculation of the residuals, and this paper uses the method proposed by Friedman [26] to calculate the residuals based on the negative gradient of the loss function.

In this paper, the negative gradient of the loss function is used as an approximation to the residuals in the boosted tree algorithm. Hence, the *i-th* sample of the m-th round *g*_*im*_ is calculated as shown in the following equation:

(10) $$\begin{array}{c} g_{im}=-{\left[\frac{\partial L\left(y_{i},f\left(x_{i}\right)\right)}{\partial f\left(x_{i}\right)}\right]}_{f\left(x_{i}\right)=f_{m-1}\left(x_{i}\right)}. \end{array}$$

*f*_*m*_(*x*) can be calculated from *β*_*m*_ and *h*_*m*_, where *β*_*m*_ denotes the optimal step for each iteration and is calculated as shown in (13). *H*_*m*_(*x*) is the decision tree created in the *m-th* iteration. The prediction is shown in (11) and (12).

(11) $$\begin{array}{c} \beta_{m}=\arg\underset{\beta }{\min}\sum_{i=1}^{n}L\left(y_{i},f_{m-1}\left(x\right)+\beta_{m}h_{m}\left(x\right)\right), \end{array}$$

(12) $$\begin{array}{c} f_{m}\left(x\right)=f_{m-1}\left(x\right)+\beta_{m}h_{m}\left(x\right). \end{array}$$

The article "Short-Term Demand Forecasting Method in Power Markets Based on the KSVM–TCN–GBRT" was published in 2022. Journal: Comput Intell Neurosci.

### 2.4. Short-Term Demand Forecasting Method Based on KSVM–TCN–GBRT

This paper takes into account day-ahead demand, real-time demand, date features, and meteorological features. An RBF kernel-SVM method is used to get the relationship between temperature, wind speed, and real-time power demand.

The TCN–GBRT method is also proposed to forecast the next day's real-time demand and the next week's real-time demand. Processing datasets are shown in Table 1.

The KSVM–TCN–GBRT method processing steps for power markets are shown in Figure 3. The short-term demand forecasting framework based on the KSVM–TCN–GBRT method is shown in Figure 4.

In this paper, parameters are selected automatically for RBFkernel-SVM by the means of temperature and wind speed. Temperature and wind speed are the main influencing factors in the new energy power market, including photovoltaic and wind power. In this paper, temperature and wind speed are proposed for measuring real-time demand class dissociative in the feature space. The same classes' temperatures and wind speeds are as close as possible. For the different classes' temperatures and wind speeds, the greater the distance that can be created between them, the better. Hence, the mean of values applied by the normal kernel function on the samples in the same class is as shown in equation (13):

(13) $$\begin{array}{c} w\left(\gamma \right)=\frac{1}{{\sum_{i=1}^{L}\left|\Omega_{i}\right|}^{2}}\sum_{i=1}^{L}\sum_{x=\Omega_{i}}\sum_{x=\Omega_{i}}\kappa \left(x,z,\gamma \right), \end{array}$$

where |Ω_*i*_| is the samples in class *i*. *β* is *w*(*γ*), which is close to 1 [29]. The RBF kernel function is as in the following equation:

(14) $$\begin{array}{c} b\left(\gamma \right)=\frac{1}{\sum_{i=1}^{L}\sum_{\begin{array}{c} j=1\\ j\neq i \end{array}}^{L}\left|\Omega_{i}\right|\left|\Omega_{i}\right|}\sum_{i=1}^{L}\sum_{\begin{array}{c} j=1\\ j\neq i \end{array}}^{L}\sum_{x=\Omega_{i}}\sum_{x=\Omega_{i}}\kappa \left(x,z,\gamma \right). \end{array}$$

Hence, *γ* should be determined such that it is closest to *b*(*γ)*. The same classes are closest to 0. The different classes are closest to 1.

It can be seen that 0 ≤ *w*(*γ*) ≤ 1 and 0 ≤ *b*(*γ*) ≤ 1 if *k*(*x*, *y*, *γ*) ≥ *t*, which is equivalent to the optimization problem, as in the following equation:

(15) $$\begin{array}{c} \underset{\beta }{\min}J\left(\gamma \right)=\left(1-w\left(\gamma \right)\right)+\left(b\left(\gamma \right)-0\right)=1-w\left(\gamma \right)+b\left(\gamma \right). \end{array}$$

In this paper, the KSVM–TCN–GBRT parameter settings are shown in Table 2.

The article "Short-Term Demand Forecasting Method in Power Markets Based on the KSVM–TCN–GBRT" was published in 2022. Journal: Comput Intell Neurosci.

Consider the impact of meteorological factors such as temperature and wind on new energy sources such as photovoltaics and wind power. In this paper, hourly datasets are extracted to create quarterly and similar day datasets based on actual electricity spot market data and weather data. This paper classifies real-time electricity demand by numerical intervals, using wind speed and temperature as the main characteristics and using 100 as the unit of measurement. A classification method using RBF SVMs with hyperparameters is used to find the optimum using numerical optimization. The wind speed and temperature are divided into groups that are particularly close to each other; the greater the difference between the different groups, the better. This master feature classification sequence is fed as a feature column into the succeeding deep learning neural network. KSVM can effectively solve machine learning problems with small samples and has good generalization ability; it can compensate for the problems of neural network structure selection and local minima.

In the electricity market, a real-time electricity demand forecast is a multivariate time series consisting of the day-ahead demand and day-ahead price. In this paper, a multivariate TCN model is developed for supervised learning, and the dynamic relationships between its variables are extracted. We take the *T* time series of the day-ahead demand and day-ahead price of the day-ahead market as the cause and the time series of real-time demand series *T* + 24 and *T* + 168 of the real-time market as the effect. By increasing the number of layers, changing the expansion coefficients, revising the filters, and adjusting the length of the historical sequence, we can avoid the gradient dispersion and gradient explosion problems in the RNN model prediction, and longer-term memory and dynamic analysis capabilities can be obtained. Also, as a convolutional structure, TCNs can slide a one-dimensional convolutional kernel to receive inputs of an arbitrary length and can be massively processed in parallel for faster training and verification. This effectively guarantees the timeliness of power prediction.

In this paper, one hot numerical treatment of meteorological features and date features is used to process the electricity market dataset into a non-high-dimensional nonsparse set of values suitable for GBRT forecasting. GBRT is integrated learning, using decision trees as weak classifiers and iterative learning based on the residuals of the decision tree predictions. It allows the GBRT model to be highly interpretative and robust, automatically discovering higher-order relationships between day-ahead market sequences and real-time demand characteristics.

The article "Short-Term Demand Forecasting Method in Power Markets Based on the KSVM–TCN–GBRT" was published in 2022. Journal: Comput Intell Neurosci.

### 2.5. Performance Evaluation

In this paper, absolute error (APE) is shown in equation (15), mean absolute percentage error (MAPE) is shown in equation (16), root mean square error (RMSE) is shown in equation (17), and mean absolute error (MAE) is shown in equation (18). The prediction errors and definitions are as follows:

(16) $$\begin{array}{c} \text{APE}=\frac{\left|P_{i}^{\text{pre}}-P_{i}^{\text{real}}\right|}{P_{i}^{\text{real}}}, \end{array}$$

(17) $$\begin{array}{c} \text{MAPE}=\frac{1}{N}\sum_{1}^{N}\frac{\left|P_{i}^{\text{pre}}-P_{i}^{\text{real}}\right|}{P_{i}^{\text{real}}}, \end{array}$$

(18) $$\begin{array}{c} \text{RMSE}=\sqrt{\frac{\sum_{1}^{N}{\left(P_{i}^{\text{pre}}-P_{i}^{\text{real}}\right)}^{2}}{N}}, \end{array}$$

(19) $$\begin{array}{c} \text{MAE}=\frac{\sum_{1}^{N}\left|P_{i}^{\text{pre}}-P_{i}^{\text{real}}\right|}{N}, \end{array}$$

where *N* is the total number of test datasets, *P*_*i*_^pre^ is the *i-th* demand prediction, and *P*_*i*_^real^ is the *i-th* demand prediction.

## 3. Results and Discussion

### 3.1. Experimental Settings

The hardware environment was Intel(R) Core(TM) i5-7200U CPU @2.70 GHz, 64 bit, 8GBDDR4 RAM memory, NVIDIA GeForce 940MX. The software development environment was Python 3.7, Tensorflow2.2.

The electricity spot market hourly dataset was obtained from ISO-NE, in the Connecticut region [27]. The meteorological data were derived from [28], and the names of weather stations were Windsor Locks and Bridgeport. The dataset spans January 1, 2016, to March 31, 2021, at an hourly frequency of 46009 moments.

The real-time demand in 2019 is shown in Figure 5. The four series of forecast dates are represented in order from top to bottom: original series, trend series, seasonal series, and residual series.

The maximum real-time demand at different temperatures is shown in Figure 6. The maximum real-time demand at different wind speeds is shown in Figure 7.

In this paper, the comparison method parameter settings are shown in Table 3.

### 3.2. Experiment 1: Real-Time Demand Forecast for the Next Day

In this experiment, the real-time power demand was predicted for a day on March 31, 2021, at an hourly frequency of 24 moments. The training dataset includes data from January 1, 2016, to March 30, 2021. The test set has data from March 31, 2020.

Real-time demand projections from March 1, 2021, to March 31, 2021, are shown in Table 4. The result of the comparison method is shown in Table 5.  Figure 8 shows the results of the KSVM-based real-time demand classification, considering the forecast results for temperature and wind speed for March 31, 2021.  Figure 9 shows the comparison between the predicted and actual demand power for each model from March 30, 2021. It can be seen that the proposed models were able to match the actual demand power in their forecasts. In particular, the proposed models could capture occasional fluctuations.

The article "Short-Term Demand Forecasting Method in Power Markets Based on the KSVM–TCN–GBRT" was published in 2022. Journal: Comput Intell Neurosci.

### 3.3. Experiment 2: Real-Time Demand Forecast for the Next Week

In this experiment, the real-time power demand was predicted for a week, from March 25, 2021, to March 31, 2021, with 168 moments. The training dataset includes data from January 1, 2016, to March 24, 2021. The test set includes data from March 25, 2021, to March 31, 2021.

The result of comparison method is shown in Table 6.  Figure 10 shows the results of the KSVM-based real-time demand classification, considering the forecasted temperature and wind speed from March 25, 2021, to March 31, 2021.  Figure 11 shows the comparison between the predicted and actual demand power for each model from March 31, 2021. It also can be seen that the proposed models were able to match the actual demand power better than other forecasts.

## 4. Conclusions

This paper proposed a novel method for short-term demand forecasting in power markets based on KSVM–TCN–GBRT. The advantages of this method over previous methods are as follows:

1. A data-driven method for short-term demand forecasting based on KSVM–TCN–GBRT was designed and improved, and the temperature and the wind speed were proposed for measuring the real-time demand to improve accuracy in forecasting market demand.
2. We adopted a model structure consisting of data classification, a time-convolutional network, and an integrated forecasting model for daily and weekly forecasts. Our proposed model can do multistep forecasting and improve the accuracy by focusing on each feature differently.
3. CNN-LSTM, LSTM with the attention mechanism, bidirectional LSTM, and TCN were used for forecasting and comparative analysis, and the operational results indicated that the proposed prediction method can reduce the prediction error and improve the prediction accuracy.

## Figures and Tables

**Figure 1:** A dilated causal convolution with dilation factors *d*=1,2,4 and filter size *k*=3.

**Figure 2:** Residual block.

**Figure 3:** The KSVM–TCN–GBRT model processing steps for Power Markets.

**Figure 4:** The short-term demand forecasting framework based on KSVM–TCN–GBRT model.

**Figure 5:** Real-time electricity demand fluctuation chart of 24 hours per day in December 2019.

The article "Short-Term Demand Forecasting Method in Power Markets Based on the KSVM–TCN–GBRT" was published in 2022. Journal: Comput Intell Neurosci.

**Figure 6:** Max real-time demand at different temperatures.

**Figure 7:** Max real-time demand at different wind speeds.

**Figure 8:** KSVM-based real-time demand classification on March 31, 2021.

**Figure 9:** Real-time demand forecast on March 31, 2021.

**Figure 10:** KSVM-based real-time demand classification from March 25, 2021, to March 31, 2021.

**Figure 11:** Real-time demand forecast from March 25, 2021, to March 31, 2021.

**Table 1:** Processing datasets.

Type of data	Input VARIABLE t	Units	Processing method	Output variable *t*
Electrical features	*t* − 24/168 day-ahead cleared demand	*MW*	https://www.iso-ne.com/ [27]	*t* + 24/168 real-time demand
	*t* − 24/168 day-ahead locational marginal price	*MW*		
		*$/MWh*		
	*t* + 24/168 day-ahead cleared demand	*MW*	*Feature extraction based on TCN*	
Meteorological feature	*t* − 24/168 temperature	*°F*	https://www.wunderground.com/ [28]	
	*t* − 24/168 dew point	*°F*		
	*t* − 24/168 humidity	*°F*		
	*t* − 24/168 wind speed	*MPH*		
	*t* − 24/168 condition	*One hot*		
	*t* + 24/168 temperature	*°F*		
	*t* + 24/168 dew point	*°F*		
	*t* + 24/168 humidity	*°F*		
	*t* + 24/168 wind speed	*MPH*		
	*t* + 24/168 condition	*One hot*		
Date features	*t* − 24/168 Week	*Day*	*Date*	
	*t* − 24/168 Month			
	*t* − 24/168 holiday			
	*t* + 24/168 Week	*Day*		
	*t* + 24/168 Month			
	*t* + 24/168 holiday			
Classification features	*t* + 24/168 classification ID		*Feature extraction based on KSVM*	

**Table 2:** the KSVM–TCN–GBRT parameter settings.

Model	Parameters	Value
Kernel SVM	Kernel	RBF
	Gamma	*γ* (automatic selecting the parameter for RBFkernel-SVM to consider temperature and wind speed)
TCN	input_channels	2
	layers_channels	[32, 16, 8, 4, 2]
	kernel_size	3
	Optimizer	Adam
	learning_rate	0.001
	Loss	mean_squared_error,
	Metrics	mse
GBRT	n_estimators	400
	Subsample	1
	min_samples_split	2
	min_samples_leaf	1
	max_depth	3
	Alpha	0.7
	learning_rate	0.2
	Loss	ls
	Verbose	0

**Table 3:** The comparison method parameter settings.

Name	Layer (type)	Output shape	Param #	Connected to
CNN- LSTM	Input (InputLayer)	[(None, 5, 2)]	0	
	conv1d (Conv1D)	(None, 5, 16)	48	input_1[0][0]
	max_pooling1d (MaxPooling1D)	(None, 1, 16)	0	conv1d[0][0]
	Dropout (dropout)	(None, 1, 16)	0	max_pooling1d[0][0]
	Dense (dense)	(None, 1，1)	17	multiply[0][0]
CNN-LSTM-attention	input (InputLayer)	[(None, 5, 2)]	0	
	conv1d (Conv1D)	(None, 5, 16)	48	input[0][0]
	max_pooling1d (MaxPooling1D)	(None, 1, 16)	0	conv1d[0][0]
	Dropout (dropout)	(None, 1, 16)	0	max_pooling1d[0][0]
	attention_vec (dense)	(None, 32)	1056	bilstm[0][0]
	Multiply (multiply)	(None, 32)	0	bilstm[0][0] attention_vec[0][0]
	Dense (dense)	(None, 1)	33	multiply[0][0]
CNN-Bi-LSTM-attention	input(InputLayer)	[(None, 5, 2)]	0	
	conv1d (Conv1D)	(None, 5, 16)	48	input[0][0]
	max_pooling1d (MaxPooling1D)	(None, 1, 16)	0	conv1d[0][0]
	Dropout (dropout)	(None, 1, 16)	0	max_pooling1d[0][0]
	Bilstm (bidirectional)	(None, 32)	4224	dropout[0][0]
	attention_vec (dense)	(None, 32)	1056	bilstm[0][0]
	Multiply (multiply)	(None, 32)	0	bilstm[0][0] attention_vec[0][0]
	Dense (dense)	(None, 1)	33	multiply[0][0]

The article "Short-Term Demand Forecasting Method in Power Markets Based on the KSVM–TCN–GBRT" was published in 2022. Journal: Comput Intell Neurosci.

**Table 4:** Real-time demand projections on March 31, 2021.

Predicted time	Actual value (MW)	CNN-LSTM		CNN-LSTM-attention		CNN-Bi-LSTM-attention		TCN		Proposed method	
		Value (MW)	APE (MW)	Value (MW)	APE (MW)	Value (MW)	APE (MW)	Value (MW)	APE (MW)	Value (MW)	APE (MW)
0: 00	2340	2697	357	2627	287	2779	439	2750	410	2348	8
1: 00	2263	2564	301	2380	117	2471	208	2527	264	2232	31
2: 00	2219	2469	250	2286	67	2369	150	2328	109	2221	2
3: 00	2204	2404	200	2282	78	2311	107	2369	165	2223	19
4: 00	2266	2360	94	2310	44	2291	25	2352	86	2266	0
5: 00	2453	2369	84	2375	78	2360	93	2520	67	2447	6
6: 00	2766	2539	227	2579	187	2571	195	2732	34	2767	1
7: 00	2996	2788	208	2889	107	2827	169	3025	29	3035	39
8: 00	3090	2950	140	3026	64	2999	91	3182	92	3093	3
9: 00	3111	3052	59	3081	30	3037	74	3245	134	3036	75
10: 00	3118	3242	124	3115	3	3111	7	3259	141	3070	48
11: 00	3090	3355	265	3093	3	3154	64	3263	173	3038	52
12: 00	3076	3409	333	3062	14	3129	53	3245	169	3013	63
13: 00	3083	3312	229	3061	22	3207	124	3236	153	3016	67
14: 00	3013	3265	252	3240	227	3218	205	3240	227	3031	18
15: 00	3004	3237	233	3151	147	3194	190	3194	190	3029	25
16: 00	3103	3134	31	3027	76	3097	6	3187	84	3054	49
17: 00	3215	3125	90	3036	179	3087	128	3253	38	3215	0
18: 00	3243	3169	74	3168	75	3146	97	3326	83	3280	37
19: 00	3252	3207	45	3218	34	3206	46	3343	91	3254	2
20: 00	3138	3209	71	3157	19	3172	34	3349	211	3146	8
21: 00	2922	3320	398	3239	317	3256	334	3258	336	2954	32
22: 00	2663	3154	491	3144	481	3127	464	2866	203	2747	84
23: 00	2441	2837	396	2803	362	2859	418	2634	193	2464	23
MAPE (%)		0.1844		0.1806		0.1876		0.1752		0.0315	
MAX APE (MW)		491		481		464		410		84	

**Table 5:** Real-time demand forecasting evaluation on the testing set.

Time	March 31, 2021		
Statistical metrics	*γ*_mae_ (MW)	*γ*_mape_ (%)	*γ*_rmse_ (MW)
CNN-LSTM	206.18	7.61	241.13
Bi-LSTM	125.56	4.66	176.31
ATT-LSTM	154.9	5.8	202.97
TCN	153.39	5.63	178.63
Proposed method	28.87	1	38.35

**Table 6:** Real-time demand forecasting evaluation on the testing set.

Time	March 25, 2021, to March 31, 2021		
Statistical metrics	*γ*_mae_ (MW)	*γ*_mape_ (%)	*γ*_rmse_ (MW)
CNN-LSTM	284.58	11.05	338.09
Bi-LSTM	216.66	8.28	279.51
ATT-LSTM	236.33	9.09	302.51
TCN	247.67	9.90	272.13
Proposed method	40.47	1.47	54.75

The article "Short-Term Demand Forecasting Method in Power Markets Based on the KSVM–TCN–GBRT" was published in 2022. Journal: Comput Intell Neurosci.

## Data Availability

The data of the models and algorithms used to support the findings of this study are included within the article.
